The article "Determination of Pesticide Residues in Food Premises Using QuECHERS Method in Bench-Sheko Zone, Southwest Ethiopia" was published in 2021. Journal: Biomed Res Int.

# Determination of Pesticide Residues in Food Premises Using QuECHERS Method in Bench-Sheko Zone, Southwest Ethiopia

**DOI:** 10.1155/2021/6612096

**Published:** 2021-03-19

**Authors:** Besufekad Mekonnen, Jafer Siraj, Samuel Negash

**Affiliations:** ^1^Department of Public Health, College of Medicine and Health Sciences, Mizan-Tepi University, Mizan-Aman, Ethiopia; ^2^School of Pharmacy, College of Medicine and Health Sciences, Mizan-Tepi University, Mizan-Aman, Ethiopia; ^3^School of Public Health, College of Medicine and Health Sciences, Mizan-Tepi University, Mizan-Aman, Ethiopia

## Abstract

Pesticides are risk factors in human life causing chronic human health effects. They are commonly used across the globe to enhance human endeavors. In Ethiopia, pesticides are widely used by local farmers and governmental organizations for pest control purpose. Pesticide residues in food items have been a concern to the consumers and environment they live in. Therefore, this study was aimed at determining the amount of organochlorine and organophosphate pesticide residues in cereal crops in Bench-Sheko Zone, Ethiopia. A cross-sectional laboratory-based study design was employed to determine the amount of pesticide residues. The samples were extracted using a Quick, Easy, Cheap, Effective, Rugged and Safe (QuEChERS) extraction and clean up method. Finally, the extracted samples were injected into gas chromatography tandem mass spectrometer and the types and concentrations of pesticide residues were analyzed. The highest concentration of endosulfan sulfate (0.076 mgkg^−1^) was detected in rice, followed by dimethoate (0.068 mgkg^−1^) and p,p′-DDE (0.087 mgkg^−1^) in sorghum and common millet, respectively, in the samples obtained from the Gurafarda site.The highest concentration of p,p′-DDT (0.133 mgkg^−1^) was detected in common millet, followed by aldrin (0.082 mgkg^−1^) and dimethoate (0.077 mgkg^−1^) in sorghum and common millet, respectively, in the samples obtained from the North Bench site. In addition, aldrin detected in rice, sorghum, and common millet obtained from the three sites was a residue of above the maximum residual limits set by Codex Alimentarius regulations and European Union. The finding shows that an indication of the widespread use of pesticides in cereal crops.

## 1. Introduction

Pesticides are poisonous chemicals intended for preventing, destroying, or controlling pests during the production, processing, transporting, and marketing of food [1, 2]. This includes vectors of human and animal diseases and unwanted species of plants or animals [3]. The use of chemicals in modern farming practices is viewed as an integral part of the success of the agricultural industry. However, most of the pesticides applied to agricultural lands may affect nontarget organisms and contaminate soil and water media [4–6]. In recent years, there has been an increasing concern that pesticides constitute a risk to the general population through residues in food supply [7].

The article "Determination of Pesticide Residues in Food Premises Using QuECHERS Method in Bench-Sheko Zone, Southwest Ethiopia" was published in 2021. Journal: Biomed Res Int.

Most pesticides used in agriculture today are synthetic organic chemicals that act by interfering with a vital metabolic process in the organisms to which they are targeted [8, 9]. The public health effects of pesticides have long been known, and the undesired effects of chemical pesticides have been recognized as a serious public health concern during the past decades [9]. According to a market survey report, approximately 5,684 million pounds of pesticides (active ingredients) are applied annually throughout the world [7]. Many of these chemicals are mutagenic and linked to the development of cancer or may lead to birth defects [10].

Genotoxic effects of malathion, cypermethrin, and carbosulfan in chromosomal aberration (sister chromatid exchange) and sperm abnormality in mice as potential germ cell were reported [6]. The health effects of pesticides can be divided into acute poisoning and chronic effects [11]. Acute pesticide poisoning is any illness or health threats appearing shortly after a single or multiple doses of pesticide [12]. This includes a wide range of reactions in different target organs like neurological, dermal, or respiratory. Chronic poisoning occurs gradually after prolonged exposure to pesticides [13]. Increasing development of cancer and reproductive abnormalities has been seen in people who exposed to pesticides for long term.

[14, 15].

A study conducted [13] on males associated with the spraying of pesticides in a farm revealed a significant increase in a chromatid breaks and gaps in chromosomes in the peripheral blood cells. However, the potential toxicity of residues still remained a matter of controversy, although it is believed that adipose tissue acts as a protective reservoir [16].

*Dichlorodiphenyltrichloroethane* (DDT) is one of the most pervasive and the persistent organic pollutant agrochemicals with widespread negative impacts on biodiversity and human health throughout the world [17]. It is taken up from the soil by plants, kills most invertebrates, particularly insects, and accumulates in the fatty tissues of animals, including humans, and leads to disruptions of normal breeding, particularly in animals that are high up the food chain such as birds of prey and in mammals that are hunters [18]. DDT is found almost everywhere in the world, even far from where it has been used as an insecticide [19].

The article "Determination of Pesticide Residues in Food Premises Using QuECHERS Method in Bench-Sheko Zone, Southwest Ethiopia" was published in 2021. Journal: Biomed Res Int.

Since the 1970s, international community through the United Nations Environment Program has been developed for controlling, or rather banning the use of DDT except under special circumstances and is known as the Stockholm Convention on persistante organic polutantes (POPs). All developed countries have now completely banned the use of DDT [7, 14, 18, 20].

Ethiopia has also developed a National Implementation Plan to eliminate or minimize the use of these chemicals. However, it is still allowed to use DDT for controlling the malaria carrying a mosquito by spraying of houses once or twice a year. These spraying campaigns are not ad hoc. They are planned to give maximum protection to people living in areas where there are regular outbreaks of malaria [5, 21].

As a result, pesticide residues in food items have been a concern to the environment and consumer groups of their widespread use [22]. Most pesticides, especially the organochlorines, are very resistant to microbial degradation. They can therefore accumulate in human body fats and the environment posing problems to human health [23–29]. In Ethiopia, from 1950s to about 2014, DDT has been sprayed outdoors (for agricultural use) as well as indoors for malaria control by reducing the density and longevity of vector mosquitoes using indoor residual spraying (IRS). Recent study done in Jimma zone shows some banned pesticides (DDT and endosulfan) were detected in the peppercorn samples [30].

Other study done in Gurage zone showed that farmers who cultivate the *Catha edulis* plant in the indicated areas of Gurage zone used DDT and spraying it on their *Catha edulis* plant to control different pests and the study revealed that the average concentrations of the first DDT metabolite, 4,4′-DDD and the second DDT metabolite, 4, 4′ of *Catha edulis* samples obtained from selected woredas of Gurage zone were higher than maximum allowable residual limits [21].

Cereal grains are the most important food grains because they are the chief source of food for the majority of the world's population. They provide about 60% of the calories and 50% of the proteins to the human race [15, 19, 26]. In Ethiopia, farmers have been widely used pesticides to achieve production efficiency in cereal crops. To date, there is no study that has been carried out to ascertain safety of cereal crops from both organochlorine and organophosphate pesticide residues. Therefore, the main objective of this study was to determine organochlorine and organophosphate pesticide residues in selected cereal crops in Bench-Sheko Zone, Ethiopia.

## 2. Materials and Methods

### 2.1. Description of the Study Area

The study was conducted in Bench-Sheko Zone. It is one of the 16 zones in South Nation Nationality regional State located 585 km away from Addis Ababa, the capital of Ethiopia, in Southwest direction. According to Ethiopia's census projection for 2014-17, in 2013E.C, the total population of the zone was786,421 out of which 388,038 were female and 398,383 were male. It has one urban and eight rural districts, 246 the smallest administrative units (229 rural and 17 urban). The zone has one University Teaching Hospital, 40 health centers and 182 health posts [31]. Geographically, Bench-Sheko Zone is located between 5°.33′ and 7°. 21′ North latitude and 34.88°′ and 36°.14′ East longitude of the equator. The zone comprises of altitudes ranging from 1200 to 1959 meters above sea level. Besides, the mean annual temperature of the zone ranges between 15 and 27°C and the mean annual rainfall ranges 1500-1800 mm [32]. According to the land utilization data of the zone, 11,383 hectares land is used for rice cultivation, 2,060 hectares for wheat production and 52‚410 hectares for corn production, 3,014.75 hectares of land is for common millet production and 18,140 hectares for sorghum cultivation [33].

The article "Determination of Pesticide Residues in Food Premises Using QuECHERS Method in Bench-Sheko Zone, Southwest Ethiopia" was published in 2021. Journal: Biomed Res Int.

### 2.2. Study Design and Period

A cross-sectional laboratory-based study design was employed to determine the types and concentration of organochlorine and organophosphate residues from selected cereal crops (rice, corn, sorghum, and common millet) in 3 major cereal crops cultivating districts (Gurafarda, South Bench, and North Bench sites) in Bench-Sheko Zone. The study was conducted from first of June to December 2019.

### 2.3. Sample Collection

The samples were collected from Bench-Sheko Zone purposively selected three sample sites, namely, Gurafarda, South Bench, and North Bench woredas (districts), where cereal crops are cultivated within the zone at large. Cereal crops (corn, sorghum, rice, and common millet) were bought from the local farms of each woreda. From each woreda again, three sites were selected. From each site, 10 samples (one kg of each crop sample) were taken randomly and homogenized to represent the bulk sample. The bulk sample of each site was placed in net polyethylene sheets until sample preparation and analysis were done [21, 30]. The data handling and measurements were carried out according to FAO and WHO Procedural Manuals [34, 35]. Moreover, sample labels were properly completed.

### 2.4. Chemicals and Reagents

All organic solvents intended for extraction were HPLC grade and purchased from different suppliers and importers found in Ethiopia. Seventeen pesticide standards were obtained from PIPARK Scientific Limited, Northampton, UK, and have analytical standard grade. These pesticide standards with their purity includes; p,p′-DDT (99%), p,p′-DDE (99.9%), chlordane (98%), hexachlor benzene (99.9%), *β*-lindane (99.5%), lindane (99.5%), *α*-lindane (99%), aldrin (97.8%), hexachlorepoxide (99.5%), *α*-endosulfan (99%), *β*-endosulfan (98.5%), endosulfan sulfate (98.8%), methoxychlor (97.7%), heptachlor (99.5%), dimethoate (98%), chlorpyrifos (99.5%), and profenofos (97.9%). All the organic solvents and reagents like acetonitrile (99.9% for HPLC), glacial acetic acid (98.5%), n-hexane (99% for HPLC), acetone (99%), magnesium sulfate (99% laboratory reagent), sodium acetate (99%), PSA (100%), and methanol (≥99.9% for HPLC) were obtained from Sigma Aldrich. Co., Germany.

The article "Determination of Pesticide Residues in Food Premises Using QuECHERS Method in Bench-Sheko Zone, Southwest Ethiopia" was published in 2021. Journal: Biomed Res Int.

### 2.5. Sample Preparation and Analysis

#### 2.5.1. Sample Extraction for Determination of Pesticides

Extraction was started with 5 g of cereal crop sample. After oven drying and grounding by mortar, 1 g of the powder was mixed with 5 ml of NaOH, sonicated for 3 minutes, and then left for 30 minutes at room temperature. Three extraction cycles were performed on the original sample with 4 ml of extraction solvent in each cycle (acetone/ethyl acetate/n-hexane (1 : 2 : 1) for three minutes vortex followed by two minutes centrifugation at 2000 g. The three extracts were combined and dehydrated with 1 g of sodium sulfate, filtered, and then reduced to 5 ml at room temperature [15, 29, 30, 34].

#### 2.5.2. QuEChERS Methods

Extraction and clean-up of the spiked samples and blank samples from each matrix were performed using the modified QuEChERS procedure with the d-SPE clean-up method [21, 30]. The procedure for spiking and extraction is as follows: (1) 5 g of comminuted and homogenized blank sample of corn, rice, common millet, and sorghum were weighed in 50 ml centrifuge tubes on an analytical balance (Sartorius); (2) 10 ml of deionized water was added; (3) blank samples were spiked with 25 ml of each pesticide standard in each matrix in 4 replicates; (4) 15 ml of acetonitrile containing 1% glacial acetic acid (*v*/*v*) in each sample was added using a solvent dispenser; (5) the tube was tightly capped and shaken gently for 1 min to facilitate contact between the solvent and the sample; (6) 6 g anhydrous MgSO4 and 1.5 g NaAc were added, and the sample was shaken by hand vigorously for 5 min to increase sample throughput; (7) the sample was centrifuged at 2016 g for 5 min; (8) for clean-up, the upper 8 ml to 10 ml were put into a d-SPE tube containing 300 mg PSA, 900 mg MgSO4, and 150 mg C18 and shaken by hand for 30 s, and then step 6 was repeated; (9) A 5 ml aliquot of cleaned extract was then taken and evaporated to dryness using a rotary evaporator (N18673 Rotavapor; Buchi) at a temperature of 40 8C; (10) the cleaned extract was reconstituted with 2 mL n-hexane:acetone (9 : 1) for solvent exchange; and (11) the extract was then put into an autosampler vial for GC analysis The sample chromatogram was evaluated against a calibration curve obtained from a 7-point calibration made using pure analytical standards for quantization purposes [21, 30].

The article "Determination of Pesticide Residues in Food Premises Using QuECHERS Method in Bench-Sheko Zone, Southwest Ethiopia" was published in 2021. Journal: Biomed Res Int.

### 2.6. Preparation of Pesticide Standards

10 mg of the pesticides standard was weighted into 10 ml biker from each and dissolved in 5 ml methanol by using ultrasonication (Elmasonic). Then, the mixture emptied into a 10 ml volumetric flask to prepare 1000 ppm stock solution. The prepared stock solution was stored in a deep freezer at -4°C. Then, the mixture emptied into a 10 ml volumetric flask to prepare 2000 ppm stock solution. From the stock solution, intermediate solution was prepared by taking 200 *μ*l from each stock solution into a 10 ml volumetric flask to prepare 20 ppm intermediate solution. A working standard was prepared by serial dilution of the Intermediate solution with n-hexane.

### 2.7. Gas Chromatography-Mass Spectroscopy (GC-MS) Conditions

Separation and determination of pesticide residues were carried out using gas chromatograph (GC-7890B manufactured by Agilent Technologies) coupled with a Triple Quadrupole Mass Spectrometer (MS-5977A model manufactured by Agilent Technologies). A DB-XLB column (60 m × 0.25 mm ID, 0.25 *μ*m film thickness, 5% phenyl methyl polysiloxane). The oven temperature was programmed initially at 60°C for 1 min, then raised to 140°C at 12°C min^−1^, and finally raised to 280°C Ag 8°C min^−1^. Pure helium was used as a carrier gas with a constant column head pressure of 50 kPa, and 1 *μ*l sample was injected in to split less injector with injection port temperature of 260°C for analysis. The mass selector detector was operated in the EI-SIM mode to determine DDT and its metabolite. The electron energy was 70 eV from the ion source, and the interface temperature was maintained at 230°C. The electron multiplier voltage was 1 kV, and the solvent delay was set to 15 min. The pesticide residues in each food sample were analyzed in triplicate, and the mean concentration was computed accordingly.

### 2.8. Analytical Method Validations

#### 2.8.1. Linearity of the Standard Curves

Calibration curves have been produced for quantification. Linearity has been observed all along the area of concentration studied depending on the target pesticide chemicals. These ranges of concentrations were selected in function of the sensitivity of the gas chromatography towards each pesticide from the correlation coefficient (*r*^2^) of the linear regression. The calibration curves were obtained by injecting eight different concentrations of the pesticide standards in a range of 4-300 ng/ml.

The article "Determination of Pesticide Residues in Food Premises Using QuECHERS Method in Bench-Sheko Zone, Southwest Ethiopia" was published in 2021. Journal: Biomed Res Int.

#### 2.8.2. Limits of Detection and Limits of Quantification

Limits of detection (LOD) and limits of quantification (LOQ) of the method were measured by spiked serial dilution of working standards prepared for calibration curves and calculated by considering a value 3 and 10 times of background noise, respectively. LOD was determined considering it as 3 times the signal to noise ratio, while LOQ was determined as 10 times the signal to noise ratio. This means that LOD and LOQ were determined as the lowest concentrations yielding a signal-to-noise (*S*/*N*) ratio of 3 and 10, respectively.

#### 2.8.3. Recovery Studies

The recovery tests were done by spiking a mixture of 17 pesticides. A pesticide standard was spiked into laboratory blank samples of corn, rice, common millet, and sorghum to give 0.25 mg/g, and recovery was based on 4 replicates. The spiked samples were left for 1 hour before extraction to allow the pesticides to partition into the matrices [30].

### 2.9. Data Analysis

The pesticides residue data was analyzed statistically using Origin Pro version 8.0 computer software packages. Analysis of variance (ANOVA) was used to assess the significance difference between the mean values of organochlorine and organophosphate pesticide residues in sample cereal crops. Possibilities less than 0.05 (*p* < 0.05) were considered statistically significant, and the analyzed data was presented by using tables [36]. All the mean values of organochlorine and organophosphate pesticide residues were compared with maximum pesticide residual limits in food samples established by Codex Alimentary and European Union standards [37, 38].

## 3. Results

A total of four cereal crops (corn, rice, common millet, and sorghum) were investigated for the presence of seventeen pesticide residues. The investigated pesticide compounds were p,p′-DDT, p,p′-DDE, chlordane, hexachlorbenzene, *β*-lindane, lindane, *α*-lindane, aldrin, hexachlorepoxide, *α*-endosulfan, *β*-endosulfan, endosulfan sulfate, methoxychlor, heptachlor, dimethoate, chlorpyrifos, and profenofos.

### 3.1. Validation Result

As presented in Table 1, the percentage recoveries of the pesticide standard were found to be acceptable ranging from 71.2% for *β*-endosulfan to 112.3% for lindane, which indicates that the reproducibility of the method was satisfactory. The limits of detection pesticides standard were ranged between 0.008 and 0.902 mgkg^−1^ and limits of quantification varied from 0.027 to 3.022 mgkg^−1^.

Calibration curves have been produced for quantification. Linearity has been observed all along the area of concentration studied depending on the target pesticide chemicals. These ranges of concentrations were selected in function of the sensitivity of the gas chromatography towards each pesticide from the correlation coefficient (*r*^2^) of the linear regression. The calibration curves were obtained by injecting eight different concentrations of the pesticide standards in a range of 4-300 ng/ml. The regression coefficient (*r*^2^) was >0.997 for all the pesticides under the study. Calibration curves of the studied analysts show satisfactory linearity over selected concentration range with regression correlation coefficients (*r*^2^) ranging from 0.997 for p,p′- DDE to 0.999 for endosulfan sulfate.

The article "Determination of Pesticide Residues in Food Premises Using QuECHERS Method in Bench-Sheko Zone, Southwest Ethiopia" was published in 2021. Journal: Biomed Res Int.

### 3.2. Analysis of Pesticide Residues

Four organochlorine pesticide residues, namely, p,p′-DDT and its metabolite (p,p′-DDE), endosulfan sulfate, and aldrin and one organophosphate pesticide residue (i.e., dimethoate) were detected from food samples collected from the sample sites. p,p′-DDT and p,p′-DDE were the most frequently detected contaminants in all food items obtained from the Gurafarda site as shown in Table 2. Pesticide residues varied from 0.011 ± 0.003 to 0.018 ± 0.005 mgkg^−1^ in corn, 0.035 ± 0.013 to 0.076 ± 0.025 mgkg^−1^ in rice, 0.037 ± 0.005 to 0.068 ± 0.042 mgkg^−1^ in sorghum, and common millet was 0.039 ± 0.030 to 0.087 ± 0.006 mgkg^−1^. Highest concentration of endosulfan sulfate (0.076 mgkg^−1^) was detected in rice (Figure 1), followed by dimethoate (0.068 mgkg^−1^) and p,p′-DDE (0.087 mgkg^−1^) in sorghum and common millet, respectively.

Table 3 illustrated that in the crop samples analyzed in the North Bench site, dimethoate was less frequently detected in corn. Highest concentration of p,p′-DDT (0.133 mgkg^−1^) was detected in common millet (Figure 2), which indicates the recent use of the pesticide DDT in the study area.

Pesticide residues varied from 0.045 to 0.066 mgkg^−1^ in corn, 0.040 to 0.077 mgkg^−1^ in rice, 0.031-0.082 mgkg^−1^ in sorghum, and 0.018-0.133 mgkg^−1^ was detected in common millet. Highest concentration of p,p′-DDT (0.133 mgkg^−1^) was detected in common millet, followed by aldrin (0.082 mgkg^−1^) and dimethoate (0.077 mgkg^−1^) in sorghum and common millet, respectively.

As illustrated in Table 4, dimethoate was detected in about 50% samples of the food items obtained from the South Bench site (Figure 3). It was only detected in rice (0.060 mgkg^−1^) and sorghum (0.051 mgkg^−1^). The average residue concentrations were varied from 0.056 to 0.059 mgkg^−1^ in corn, 0.035 to 0.057 mgkg^−1^ in rice, 0.051 to 0.130 mgkg^−1^ in sorghum, and 0.038 to 0.074 mgkg^−1^ in common millet. Highest concentration of the aldrin residue (0.130 mgkg^−1^) was detected in sorghum (Figure 4).

The article "Determination of Pesticide Residues in Food Premises Using QuECHERS Method in Bench-Sheko Zone, Southwest Ethiopia" was published in 2021. Journal: Biomed Res Int.

### 3.3. Comparison of Pesticide Residue with the Maximum Residue Limit (MRL)

Tables 5–7 summarize the comparison of average mean concentration of detected residues with MRLs established by the European Union (EU) and the Codex Alimentarius regulations. As indicated in Table 5, the comparisons of residue concentration in food samples obtained from the Gurafarda site are as follows: aldrin was detected in rice, sorghum, and common millet where the residue was above the MRLs set by Codex Alimentarius regulations [39] and European Union (EU) [40], while the dimethoate residue detected in rice, sorghum, and common millet contained a residue of above the MRLs set by European Union(EU). In addition, p,p′-DDT in common millet and endosulfan sulfate in rice abide by the corresponding MRLs set by EuropeanUnion.

The average concentration of p,p′-DDT and p,p′-DDE residues detected in all food samples obtained from the North Bench site was above the MRLs established by the European Union and p,p′-DDT and endosulfan sulfate residues detected in common millet and rice were also above the MRLs established by Codex Alimentarius standards and European Union, respectively, as shown in Table 6. The average concentration of aldrin residue detected in all food samples obtained from this site was above the MRLs established by Codex Alimentarius standards and European Union. The only organophosphate (dimethoate) detected in three food samples (i.e., rice, sorghum, and common millet) obtained from the North Bench site was also above the MRLs established by European Union.

The average concentration of p,p'′-DDT and p,p′-DDE residues detected in all food samples obtained from the South Bench site were above the MRLs established by the European Union as indicated in Table 7. Moreover, endosulfan sulfate residue was detected in three food items, namely, corn, rice, and sorghum. It was above the MRLs established by the European Union. The average concentration of aldrin residue detected in all food samples obtained from this site was above the MRLs established by Codex Alimentarius standards and European Union. Dimethoate residue detected in 50% of the food sample was above the MRLs established by the European Union.

## 4. Discussion

In the present study, four organochlorine pesticide residues, namely, p,p′-DDT and its metabolite (p,p′-DDE), endosulfan sulfate, and aldrin and one organophosphate pesticide residue (i.e., dimethoate) were detected in food samples collected from sample sites. p,p′-DDT and p,p′-DDE were the most frequently detected contaminants in all food items. The chlorinated pesticides such as DDT and endusulfan are mostly used for malaria control in Ethiopia [5, 21]. This might be due to cross contamination or from their persistent nature remain in the nearby environment [29].

The article "Determination of Pesticide Residues in Food Premises Using QuECHERS Method in Bench-Sheko Zone, Southwest Ethiopia" was published in 2021. Journal: Biomed Res Int.

In this study, p,p′-DDT and p,p′-DDE residues were detected in all food samples obtained from the three sites. This could be due to pesticides with high volatility can be absorbed by the foliar of nontarget crops through spray drift and can also be taken up by crop roots under dry soil conditions [41]. One other possible way by which the contamination could arise is through contaminated surfaces due to storage and distribution practices. The result of the present study is consistent with a study done in Jimma zone (Ethiopia) which reported that the concentration of DDT in coffee pulp is significantly differed (*p* value < 0.01) from other food items except for red pepper [30]. Although DDT is officially banned for agricultural application in Ethiopia, contamination of food still occurs. This contamination might be explained by indoor spraying of DDT for malaria prevention and by illegal use from obsolete pesticide stocks [5, 21, 30]. In addition, it might be due to persistent nature of organochlorine pesticides prevail in the nearby soil and water compartment [29].

The only organophosphate (dimethoate) was detected in corn obtained from the sample sites. This is due to the fact that organophosphate compounds have the advantage of being more rapidly degraded in the environment than organochlorine compounds [6]. Generally, dimethoate residue was less frequently detected in all food items obtained from the three sites and above the MRL of cereals established by the European Union [39, 42].

The commonly consumed food items in Bech-Maji zone shows lower concentrations of p,p′-DDT pesticide residues except the p,p′-DDE residue was of higher concentration reported from Jimma zone, Ethiopia [30]. This variation could be attributed to the fact that Jimma zone is a high potential area in agriculture and there is a possibility of organochlorine pesticide use in the past. Additionally, higher residues may result from historical use and previous environmental contamination, particularly from those compounds demonstrating environmental persistence and accumulation of obsolete pesticides nearby the study area [5].

The comparisons of residue concentration in food samples obtained from Gurafarda showed that aldrin detected in rice, sorghum, and common millet were above the MRLs set by Codex Alimentarius regulations [39] and European Union [40], while the dimethoate residue detected in rice, sorghum, and common millet were contained above the MRLs set by European Union (EU). In addition, p,p′-DDT in common millet and endosulfan sulfate in rice exceeded corresponding MRLs set by the European Union [40].

The article "Determination of Pesticide Residues in Food Premises Using QuECHERS Method in Bench-Sheko Zone, Southwest Ethiopia" was published in 2021. Journal: Biomed Res Int.

The average concentration of p,p′-DDT and p,p′-DDE residues detected in all food samples obtained from the North Bench site were above the MRLs established by the European Union and p,p′-DDT and endosulfan sulfate residue detected in common millet and rice were also above the MRLs established by Codex Alimentarius standards and European Union, respectively. Similar result reported when compared to the study done in Jimma zone, Ethiopia, which showed that DDT which was expressed as the total sum of its metabolites: p,p′-DDE, p,p′-DDD, o,p′-DDT, and p,p′-DDT, was above the MRL set by Codex Alimentarius [40] in the two commonly consumed cereals corn and teff. The reason might be due to illegal use of pesticides in the production of staple crops in the study area or there may be contamination from the environment [30].

### 4.1. Estimated Daily Intake (EDI) of Pesticides in Food

The Joint Food and Agriculture Organization of the United Nations FAO/WHO Codex Alimentarius Commission have set the acceptable daily intake (ADI) for total DDT, endosulfan sulfate, aldrin and dimethoate to be 0.01 mgkg^−1^, 0.006 mgkg^−1^, 0.0001 mgkg^−1^, and 0.002 mgkg^−1^, respectively [43]. The ADI is explained based on a body weight of a person who utilizes pesticide residues individually may be exposed daily over his or her lifetime without appreciable health risk [43]. In order to know the exposure of consumers of pesticide residues, the estimated daily intake (EDI) of these pesticides was determined from the measured concentrations. Human health risk estimations were done based on the pesticide residue database and cereal crop consumption assumptions per capita per year, and by considering 60 kg as average body weight. The annual consumption of corn, rice, sorghum, and common millet were 18.864 kg/person/year, 58.164 kg/person/year, 4.716 kg/person/year, and 3.144 kg/person/year, respectively [44]. Results obtained were used to calculate EDI and expressed as microgram pesticides per kilogram body weight per day (mg/kg bw/day) (Table 8).

The EDI is a realistic estimate of pesticide exposure that was calculated for each pesticide in cereal crops in agreement with the international guidelines [45], using the following equation:

(1) $$\begin{array}{c} \text{EDI}=\Sigma C\times \frac{\text{F}}{\text{D}}\times W, \end{array}$$

where *C* is the mean concentration of the pesticide in cereal crops (mgkg^−1^), *F* is mean annual intake of cereal crops per person, *D* is number of days in a year (365), and *W* is mean body weight (60 kg).

The article "Determination of Pesticide Residues in Food Premises Using QuECHERS Method in Bench-Sheko Zone, Southwest Ethiopia" was published in 2021. Journal: Biomed Res Int.

According to the current study, the EDI of total DDT ranges from 0.17 to 0.56 mgkg^−1^ which is higher than the range recommended by the FAO/WHO ADI value. Also, estimated daily intakes of endosulfan sulfate, aldrin, and dimethoate were greater than ADIs which shows that cereal crops consumers are exposed to these chemicals above the limit.

## 5. Conclusion and Recommendations

Four cereal crops were investigated for the presence of pesticide residues. Out of them, only five pesticide residues were detected. Four organochlorine pesticide residues, namely, p,p′-DDT and its metabolite (p,p′-DDE), endosulfan sulfate, and aldrin and one organophosphate pesticide residue (i.e., dimethoate) were detected in food samples collected from the three areas. p,p′-DDT and p,p′-DDE were the most frequently detected contaminants in all food items obtained from the Gurafarda and North Bench sites. Dimethoate was detected in 50% samples of the food items obtained from the South Bench site.

Tighter regulation in the production of cereal crops and implementation of integrated pest management methods should be needed. Additionally, further monitoring studies must be performed to improve food safety and protect consumers' health. In Ethiopia, there is no maximum residue limit set by the concerned bodies. Therefore, establishment of the national maximum residue limits is recommended. In addition, the use of organophosphate and organochlorine pesticides are common in cereal crop production; hence, monitoring of this chemicals should be done at regular interval to determine the extent of the release of these compound's to environmental compartment and food products. Moreover, strict regulations on this pesticides and also further monitoring should be implemented that dietary pesticide exposures from other food products such as vegetables, fruits, dairy, fish, and meat should be investigated and cumulative risk assessment should be done from collective consumption. As such, estimates are not considered total dietary exposure to the pesticides, nor do we consider drinking water, residential, or occupational exposures.

## Figures and Tables

**Figure 1:** Sample chromatogram for endosulfan sulfate residues.

**Figure 2:** Sample chromatogram for p,p′-DDT residues.

**Figure 3:** Sample chromatogram for dimethoate residues.

**Figure 4:** Sample chromatogram for aldrin residues.

**Table 1:** Percentage recoveries and validation information of pesticide standards used for this study.

Pesticide standard	Percentage recovery (%)	Limits of detection (mgkg^−1^)	Limits of quantification (mgkg^−1^)
			
p,p′-DDE	90.5	0.010	0.033
p,p′-DDT	85.7	0.016	0.054
Chlordane	101.6	0.108	0.362
Endosulfan sulfate	72.4	0.008	0.027
*α*-Endosulfan	98.1	0.078	0.261
Hexachlor benzene	81.3	0.241	0.807
*β*-Lindane	73.9	0.512	2.705
Lindane	112.3	0.016	0.054
*α*-Lindane	82.3	0.193	0.647
Aldrin	89.4	0.020	0.067
Hexachlorepoxide	78.8	0.902	3.022
Methoxychlor	91.2	0.038	0.127
Heptachlor	81.4	0.193	0.647
Dimethoate	94.8	0.018	0.060
Chlorpyrifos	88.0	0.310	1.039
Profenofos	71.5	0.032	0.107
*β*-Endosulfan	71.2	0.205	0.687

The article "Determination of Pesticide Residues in Food Premises Using QuECHERS Method in Bench-Sheko Zone, Southwest Ethiopia" was published in 2021. Journal: Biomed Res Int.

**Table 2:** Concentration (mgkg^−1^) of pesticide residues in assessed food items from the Gurafarda site.

Pesticide residues	Food items			
	Corn	Rice	Sorghum	Common millet
p,p′-DDT	0.018 ± 0.005	0.046 ± 0.020	0.048 ± 0.007	0.062 ± 0.027
p,p′-DDE	0.011 ± 0.003	0.035 ± 0.013	0.054 ± 0.009	0.087 ± 0.006
Endosulfan sulfate	ND	0.076 ± 0.025	0.047 ± 0.013	0.039 ± 0.030
Aldrin	ND	0.06 ± 0.033	0.037 ± 0.005	0.042 ± 0.008
Dimethoate	ND	0.065 ± 0.023	0.068 ± 0.042	0.080 ± 0.018

**Table 3:** Concentration (mgkg^−1^) of pesticide residues in assessed food items from the North Bench site.

Pesticide residues	Food items			
	Corn	Rice	Sorghum	Common millet
p,p′-DDT	0.064 ± 0.023	0.059 ± 0.26	0.031 ± 0.011	0.133 ± 0.069
p,p′-DDE	0.066 ± 0.039	0.058 ± 0.027	0.044 ± 0	0.057 ± 0.007
Endosulfan sulfate	0.045 ± 0.003	0.061 ± 0.034	0.049 ± 0.018	0.018 ± 0.002
Aldrin	0.065 ± 0.028	0.040 ± 0.02	0.082 ± 0.007	0.027 ± 0.002
Dimethoate	ND	0.077 ± 0.028	0.04 ± 0.013	0.039 ± 0.006

**Table 4:** Concentration (mgkg^−1^) of pesticide residues in assessed food items from the South Bench site.

Pesticide residues	Food items			
	Corn	Rice	Sorghum	Common millet
p,p′-DDT	0.056 ± 0.042	0.035 ± 0.013	0.075 ± 0.022	0.038 ± 0.016
p,p′-DDE	0.059 ± 0.023	0.057 ± 0.023	0.078 ± 0.018	0.074 ± 0.022
Endosulfan sulfate	0.081 ± 0.004	0.065 ± 0.023	0.059 ± 0.036	0.044 ± 0.020
Aldrin	0.074 ± 0.025	0.069 ± 0.027	0.130 ± 0.146	0.045 ± 0.017
Dimethoate	ND	0.060 ± 0.030	0.051 ± 0.021	ND

**Table 5:** Comparisons of average mean concentration of pesticide residues with European Union and Codex Alimentareous standards from the Gurafarda site.

Pesticide residues	Food items											
	Corn	MRLs		Rice	MRLs		Sorghum	MRLs		Common millet	MRLs	
		CA	EU		CA	EU		CA	EU		CA	EU
p,p′-DDT	0.018	0.1	0.05	0.046	0.1	0.05	0.048	0.1	0.05	0.062	0.1	0.05
p,p′-DDE	0.011	0.1	0.05	0.035	0.1	0.05	0.054	0.1	0.05	0.087	0.1	0.05
Endosulfan sulfate	ND	NA	0.05	0.076	NA	0.05	0.047	NA	0.05	0.039	NA	0.05
Aldrin	ND	0.02	0.01	0.06	0.02	0.01	0.037	0.02	0.01	0.042	0.02	0.01
Dimethoate	ND	NA	0.01	0.065	NA	0.01	0.068	NA	0.01	0.080	NA	0.01

MRLs: maximum residue limits; NA: not available; ND: not detected; CA: Codex Alimentarius; EU: European Union.

**Table 6:** Comparisons of average mean concentration of pesticide residues with European Union and Codex Alimentareous standards from the North Bench site.

Pesticide residues	Food items											
	Corn	MRLs		Rice	MRLs		Sorghum	MRLs		Common millet	MRLs	
		CA	EU		CA	EU		CA	EU		CA	EU
p,p′-DDT	0.064	0.1	0.05	0.059	0.1	0.05	0.031	0.1	0.05	0.133	0.1	0.05
p,p′-DDE	0.066	0.1	0.05	0.058	0.1	0.05	0.044	0.1	0.05	0.057	0.1	0.05
Endosulfan sulfate	0.045	NA	0.05	0.061	NA	0.05	0.049	NA	0.05	0.018	NA	0.05
Aldrin	0.065	0.02	0.01	0.040	0.02	0.01	0.082	0.02	0.01	0.027	0.02	0.01
Dimethoate	ND	NA	0.01	0.077	NA	0.01	0.04	NA	0.01	0.039	NA	0.01

MRLs: maximum residue limits; NA: not available; ND: not detected; CA: Codex Alimentarius; EU: European Union.

The article "Determination of Pesticide Residues in Food Premises Using QuECHERS Method in Bench-Sheko Zone, Southwest Ethiopia" was published in 2021. Journal: Biomed Res Int.

**Table 7:** Comparisons of average mean concentration of pesticide residues with European Union and Codex Alimentareous standards from the South Bench site.

Pesticide residues	Food items											
	Corn	MRLs		Rice	MRLs		Sorghum	MRLs		Common millet	MRLs	
		CA	EU		CA	EU		CA	EU		CA	EU
p,p′-DDT	0.056	0.1	0.05	0.035	0.1	0.05	0.075	0.1	0.05	0.038	0.1	0.05
p,p′-DDE	0.059	0.1	0.05	0.057	0.1	0.05	0.078	0.1	0.05	0.074	0.1	0.05
Endosulfan sulfate	0.081	NA	0.05	0.065	NA	0.05	0.059	NA	0.05	0.044	NA	0.05
Aldrin	0.074	0.02	0.01	0.069	0.02	0.01	0.130	0.02	0.01	0.045	0.02	0.01
Dimethoate	ND	NA	0.01	0.060	NA	0.01	0.051	NA	0.01	ND	NA	0.01

MRLs: maximum residue limits; NA: not available; ND: not detected; CA: Codex Alimentarius; EU: European Union.

**Table 8:** Estimated daily intakes (EDIs) of pesticide residues detected in cereal crops.

Pesticide residues	EDIs (mg/kg bw/day)											
	Corn			Rice			Sorghum			Common millet		
	GFs	NBs	SBs	GFs	NBs	SBs	GFs	NBs	SBs	GFs	NBs	SBs
p,p′-DDT	0.06	0.17	0.17	0.44	0.56	0.33	0.03	0.02	0.06	0.03	0.07	0.02
p,p′-DDE	0.03	0.20	0.18	0.33	0.55	0.54	0.04	0.03	0.06	0.04	0.03	0.04
Endosulfan sulfate	ND	0.14	0.25	0.73	0.58	0.62	0.03	0.04	0.04	0.02	0.01	0.02
Aldrin	ND	0.20	0.23	0.57	0.38	0.66	0.03	0.06	0.10	0.02	0.01	0.02
Dimethoate	ND	ND	ND	0.62	0.73	0.57	0.05	0.03	0.04	0.04	0.02	ND

Key: EDIs: estimated daily intakes; GFs: Gurafarda site; NBs: North Bench site; SBs: South Bench site.

## Data Availability

All data are available based on reasonable request.

## Abbreviations

ADI: Acceptable daily intake
CA: Codex Alimentarius
DDT: Dichlorodiphenyltrichloroethane
EDIs: Estimated daily intakes
EU: European Union
MRLs: Maximum residue limits
NA: Not available
ND: Not detected
OC: Organochlorine
OP: Organophosphate
POPs: Persistent organic pollutants
PSA: Primary and secondary amine
QuEChERS: Quick, easy, cheap, effective, rugged and safe
WHO: World Health Organization.

## Additional Points

- Four organochlorine pesticide residues, namely, p,p′-DDT and its metabolite (p,p′-DDE), endosulfan sulfate, and Aldrin, and one organophosphate pesticide residue (i.e., Dimethoate) were detected in the study area
- p,p′-DDT and p,p′-DDE were the most frequently detected contaminants in all food items
- The ratio of DDT to DDE has indicated the persistent use of DDT in the area
- Dimethoate was detected in 50% samples of the food items obtained from South Bench site
